RETRACTED

# Development of Health Digital GIS Map for Tuberculosis Disease Distribution Analysis in Sudan

**DOI:** 10.1155/2023/6479187

**Published:** 2023-02-13

**Authors:** Mohamed Sidahmed M. Siddik, Thowiba E. Ahmed, Fatima Rayan Awad Ahmed, Rania A. Mokhtar, Elmustafa Sayed Ali, Rashid A. Saeed

**Affiliations:** ^1^Faculty of Computer Science and Information Technology, Al Neelain University, Khartoum, Sudan; ^2^Computer Science Department, College of Science and Humanities-Jubail, Imam Abdulrahman Bin Faisal University, Jubail 35811, Saudi Arabia; ^3^Computer Science Department, College of Computer Engineering and Science, Prince Sattam Bin Abdulaziz University, Al-Kharj 11942, Saudi Arabia; ^4^Computer Engineering Department, College of Computers and Information Technology, Taif University, P.O. Box 11099, Taif 21944, Saudi Arabia; ^5^Electrical and Electronics Engineering Department, Faculty of Engineering, Red Sea University, Port-Sudan, Sudan; ^6^Electronics Engineering School, College of Engineering, Sudan University of Science and Technology (SUST), Khartoum, Sudan

## Abstract

Health digital GIS map provides a great solution for medical geographical distribution to efficiently explore diseases and health services. In Sudan, tuberculosis disease is expanding in different areas, which requires a digital GIS map to collect information about the patients and support medical institutions by geographical distribution based on health services, drug supply, and consumption. This paper developed a health digital GIS map to provide a fair geographical distribution of tuberculosis health centers and control the drug supply according to medical reports. The proposed approach extracts the unfair distribution of medicine, as some centers receive medicine but do not receive patients, while others receive a large number of patients but limited amounts of medicine. The analysis results show that there is a defect in some states representing the distribution of tuberculosis centers. In the Northern State, there are 15 tuberculosis centers distributed over all localities, serving about 84 tuberculosis-infected patients only.

## 1. Introduction

Geography is a science that emerged with the existence of human beings on the Earth attempting to explore the characteristics and features of the place we are living. With the advent of the information revolution, geography plays an important role in the integration of information technology with various applications related to geographical sciences [1]. Geography has been branched into so many subspecialized sciences, one of the most reputed being “medical geography” or “health geography” [2].

The great importance of medical geography is derived from its ability to mix advanced geographical technologies with health information to study the health situation and explore the efficiency of the geographical distribution of health services. The digital geographic information system (GIS) technology allows for the efficient acquisition, management, processing, and analysis of distributed medical and health data. The diseases and medical reports in a country can be analyzed to obtain the current condition of medical issues and the distribution of hospitals and drugs as well.  Figure 1 shows the schematic diagram of a digital GIS map.

RETRACTED

Sudan is located in the middle part of the Nile valley, located on the latitudes 8.45–22.8 and longitudes 21.49–38.34 [3], it occupies a central location between Africa and the Middle East, with an area estimated at 1,865,813 square kilometers, ranking as the 3rd largest land area in Africa after Algeria and Democratic Republic of Congo, and 16^th^ largest country in the world.

Sudan borders seven African countries, which are Egypt, Libya, Eritrea, Ethiopia, Chad, the Central African Republic, and the Republic of South Sudan [4]. Most of the countries bordering Sudan are suffering from the burden of poverty, armed conflicts, and civil wars [5]. The people of these countries are classified below the poverty line according to the annual World Bank reports [6]. The total population of Sudan is estimated at 33,419,652 persons, occupying the 38^th^ rank in the world and the 9^th^ rank in Africa [7].

According to the sources reviewed by the researchers during their interviews, the relationship between Sudan and tuberculosis dates back to the Turkish period, when some of the Sudanese soldiers were sent abroad to fight among the ranks of the Turkish fighting groups [8]. They brought tuberculosis infection when they returned to Sudan. This is supported by the fact that no single case had been reported in Sudan before 1885, despite the spread of other infectious diseases such as sleeping sickness and cholera. The objective of this research is to tackle the creation of a digital GIS map for tuberculosis disease in Sudan by using the GIS connected with the databases that link the data with its spatial location [9].

The aim of this paper is to describe the development of a digital GIS map for TB disease analysis in Sudan which will provide a fair geographical distribution of tuberculosis health centers and control the drug supply according to medical reports.

The remainder of the paper is organized as follows: Section 2 presented the problem statement and formulation.  Section 3 presented related works. In Section 4, the material and methods were presented. In Section 5, the results and discussion were discussed. In Section 6, the paper is concluded and some recommendations and future works were stated.

RETRACTED

## 2. Problem Formulation and Statement

Transmitted diseases are considered a difficult health problem that poses a threat to a large part of the population. Recently, GIS has been used in many applications, such as natural resource management and agriculture. Recently, institutions have turned to using GIS to assess and model the relationships between environmental factors and cases of viral diseases [10]. In Sudan, a number of diseases such as cholera, dysentery, and tuberculosis are considered as the most serious threat to human health and the economy. The use of GIS and remote sensing enables to provide a comprehensive system of public health care and epidemiology.

At present, tuberculosis is spread all over Sudan without exception, and unfortunately, the highest infection rates are in the capital, Khartoum, between productive age groups from age 15 to 44 [11, 12].  Table 1 shows the number of tuberculosis cases in Sudan during the year 2013, according to the World Health Organization (WHO) report [13].

Medicine consumption is a human phenomenon that lasts as long as life exists, and it will be far away from market theories, which are based on supply and demand; medicines are never liable to postponement or waiting regardless of the patient's place or economic condition [14]. The problems, which this study attempts to explore and reach acceptable solutions, are summed up in the following:

- The absence of a digital map for tuberculosis disease in Sudan shows clearly the real number of TB patients in Sudan and their geographical location, as well as the quantity of circulated medicine and the relationship between this disease and different demographic factors [15].
- The absence of a geographic database for the health sector and its institutions concerned with the treatment of tuberculosis in Sudan.

## 3. Related Works

The geographical information system is a computerized system for capturing, managing, and processing spatial data. The spatial means the geographical features on the Earth's surface or any other industrial features such as buildings, roads, or other natural phenomenon features [16]. The GIS is used in the process of planning and supporting strategic decisions and policy-making. Researchers defined the GIS from a geographical and technical perspective as a mixture of geographic data and cognitive expertise of the geographical experts and the modern digital technologies that have greatly contributed to the development and upgrading of human life as an effective tool for collecting information, storage, processing, analysis, and displaying the results in different ways depending on the desired goal.

RETRACTED

Kurland [17] reviewed the research of geographical patterns of diseases as an important support for the investigation of outbreaks; analyzing the geographic nature of disease cases has been a key factor in finding out the source of many outbreaks.

In [18], Koch provides that the field of medical geographic information systems (medical GIS) has become extremely useful in understanding the bigger picture of public health. The discipline holds a substantial capacity to understand not only differences but also similarities in population health around the world.

Oirba in [19] presented radar data for the main valleys of all the rivers that were mapped and contrasted with those identified by the hydrological GIS procedures. In the past, the banks of these river courses, which are now devoid of groundwater, may have hosted a substantial amount of available water and played an important role in recharging the region's natural stone groundwater aquifers.

In [20], a new technique that has been developed for determining the preliminary optimal general position of the route using GIS is discussed. There are two key phases of the established process. In the first step, using effective contour (snakes) algorithms based on satellite picture gray values, an initial set of required action locations is independently optimized [21]. Linear programming (LP) is used by the built (path tools) as an evolutionary algorithm to calculate an overall provisional optimal route position using a rough estimate based on three factors: distance traveled of the route, levels of the route section, and degree of curvature between conditions required of the route.

In [22], a GIS of tuberculosis in Mombasa County in 2015–2017 is discovered in the study. The paper employed a survey approach acquired from government secondary data. The community was registered at 30 centers for all patients suspected of having tuberculosis, and the measurements were done by tuberculosis clinicians with phlegm (+) and (−) exams.

According to Musa et al. in [23], the main goal was to examine the spatial distribution of TB cases in Kuala Lumpur municipal area and recognize spatial trends. A location GIS map was used to highlight the high-risk and spatial areas of the TB outbreak in KL. Mean K-nearest distance and spatial autocorrelation spatial statistical methods were also used.

In [24], research on a business model for the advancement of medical techniques in the Soviet Union for the period leading up to 2025 is conducted. With the support of applied resources, it is clear that it is necessary to stimulate the growth of phthisiology in particular and to improve the efficacy of the use of the findings in the clinical and institutional treatment of antituberculosis and associated Russian organizations [25].

RETRACTED

## 4. Material and Methodologies

The methodology is based on data collection on the TB medicine consumption at Sudanese states, municipalities, specialized tuberculosis treatment centers, and then field work to cover the shortfall of unavailable information. This shall be done through a remote sensing technique and predictions through four phases as shown in Figure 2.

### 4.1. Data Collections

We collected the available data from its basic sources, the Federal Ministry of Health [26], Central Medical supply [27], National Medicines and Poisons Board [28], National Medical Supplies Fund [29], United Nations Development Program, Sudan [30], and National TB Control Program, Sudan [31]. These data helped researchers for general understanding and created a fundamental perception of the number of TB patients who take regular treatment, disease linkage with the location, and assessing the effectiveness of the TB control program, and then researchers linked these data with the location data, which include the following:

- Topographic maps for each state scale 1100.000
- Improved satellite images, ETM + 7 type [32], and eight optical bundles of 15-meter accuracy
- High accuracy images, 0.61 meters, for cities where health services are available in each state, Quickbird type in addition to radar images
- Sudan map, scale 1100.000 [33]

### 4.2. Remote Sensing Data

We used remote sensing and GIS data for map drawing from extracted satellite images. The GIS was used as a spatial data visualization tool to help develop a model to study all potential scenarios for the relation between TB medicine consumption and a number of infected persons in the area. 

Maps, images, and other data shall be interpreted by linking drug distribution and consumption with spatial and temporal data to benefit from the GIS capacities to provide the best method to combine the various types of data to produce a map that supports the decision-makers on the actual health level to contribute in achieving the efforts in all health sectors, international organizations, and civil community organizations to defeat this disease.

### 4.3. Descriptive and Interpretational Data

The descriptive and interpretational data in the first and second stages are liable to statistical analysis at this stage, the outputs of which are the main source of the target database through this research. This phase also contains the mapping of all health facilities providing tuberculosis treatment in Sudan.

RETRACTED

### 4.4. Data Analysis

The analyzed data contain information related to the distribution of hospitals and health centers specialized in TB treatment. The researcher has used the GIS ARC 10.3 application to represent the (X, Y) coordinates of the health centers concerned with the TB treatments, which we are working on in 11 states out of 17 states. The researcher failed to make field visits to the remaining states because they are unstable due to security issues. ArcGIS is an analysis and mapping solution based on online cloud. Researchers are utilizing it to illustrate and represent data, analyse, collaborate, and share map-based data. GIS ARC 10.3 has the capability to access workflow-specific applications, data, and maps from around the world and is a tool for being shared and collaborated on in the area of this research [34].

Through an analysis of the obtained information and based on the population census of each state, the researcher has discovered the defect in some states representing the distribution of tuberculosis centers, for example, the Northern State has 15 tuberculosis centers distributed over all localities serving about 84 tuberculosis-infected patients only (Figures 3–5).

### 4.5. GIS Reports

One of the main objectives of this study is to provide accurate reports helping the decision-makers by making available the required figures and information based on and extracted by scientific methods [35]. Therefore, we find out that the system has provided the stakeholders and concerned authorities with the possibility of accessing the system site through the Internet and generating the required reports based on the processed data. Figures 6–8 are reports showing the number of tuberculosis-infected persons in each state compared with the existing population of the state, distribution of patients, and distribution of drugs.

## 5. GIS Database Results and Discussion

The geographic database for the health sector and its institutions concerned with the treatment of tuberculosis includes (339) specialized centers for examination and treatment of tuberculosis revealed as shown in Table 2 and Figure 9. The results of the distribution of tuberculosis drugs to the health institutions concerned with the treatment of the disease are shown in Table 3.

Sudan belongs to a third-world country that receives humanitarian aid from donor countries, and because of corruption and lack of scientific information and proper planning, most of these aids do not reach those who need them, especially in the health field.

The results of the research showed that there is an unfair distribution of medicine, as some centers receive medicine but do not receive patients. On the contrary, some centers receive a large number of patients and limited amounts of medicine, which can benefit from the quantities of drugs distributed randomly. Unfortunately, the World Health Organization (WHO) has announced the closure of several health centers due to a lack of funds and an increase in the number of displaced and affected people in conflict areas, although the research showed that there is a surplus in drug resources.

RETRACTED

## 6. Conclusion

Therefore, this research tackles the creation of a digital map for tuberculosis disease in Sudan by using the GIS to connect it with the databases, namely, linking the data with its spatial location. According to this research, we recommend the following: Firstly, the researcher recommends studying the relationship among TB disease, economic conditions, and the national income of the tuberculosis patients' areas since the researcher has noticed the spread of the disease in poor and densely populated areas, a matter that will aggravate the health situation. The researcher adopted equally fair distribution of specialized TB centers over the country by using the geographic information systems for tracking and monitoring the places where the patients are found for a fair distribution of the drug and by using the geographic information systems to contribute to the improvement of health systems and provide a real picture of the nature and spread of the disease.

## Figures and Tables

**Figure 1:** Schematic diagram of the GIS digital map.

**Figure 2:** Development of digital GIS map for tuberculosis disease analysis phases.

**Figure 3:** Distribution of tuberculosis centers in the Northern State.

**Figure 4:** Distribution of tuberculosis patients in Northern State.

**Figure 5:** Distribution of tuberculosis drugs in Northern State.

**Figure 6:** Comparison between states according to the number of patients.

**Figure 7:** Distribution of patients.

**Figure 8:** Distribution of drugs.

**Figure 9:** Number of centers that received patients.

**Table 1:** Total number of TB patients undergoing treatment through the National Tuberculosis Control Program.

Year	New cases	Sputum positive cases	Sputum negative cases	Extrapulmonary TB	No of HIV/TB
2010	47,643	9958	9144	6217	7532
2011	42,348	7266	6746	4624	3082
2012	41,775	6587	6948	4561	3070
2013	40,388	7708	6088	4915	3056
2014	37,392	9734	6106	4571	3762
2015	35,006	9888	6190	4578	3789
2017	30,674	9912	6671	4708	3811
2018	28,410	10002	7201	4850	3899
2019	26,801	10272	8698	4901	4016
2020	25,215	10453	8761	5409	4112

**Table 2:** Number of centers that received patients.

No.	No. of centers	Patients
1	111	0
2	148	50
3	33	50 to 100
4	14	100 to 150
5	15	150 to 200
6	3	200 to 250
7	4	350 to 400
8	4	400 to 450
9	4	450 to 500
10	2	500 to 550
11	2	600 to 650
12	One center in the capital city of Khartoum	**2544**

This value represents the patients in Khartoum city. The bold does not make additive sense to the value but is used just to indicate the largest number of patients.

RETRACTED

**Table 3:** The results of the distribution of tuberculosis drugs to the health institutions concerned with the treatment of the disease.

	No. of centers	Tuberculosis drug availability
1	59	Tuberculosis drugs received but they received no patients
2	13	282 tuberculosis patients did not receive drug

## Data Availability

The datasets and codes generated during and/or analyzed during the current study are available from the corresponding author on reasonable request.
